The article "Ethnopharmacological Study of Medicinal Plants in Bajwat Wildlife Sanctuary, District Sialkot, Punjab Province of Pakistan" was published in 2021. Journal: Evid Based Complement Alternat Med.

# Ethnopharmacological Study of Medicinal Plants in Bajwat Wildlife Sanctuary, District Sialkot, Punjab Province of Pakistan

**DOI:** 10.1155/2021/5547987

**Published:** 2021-10-25

**Authors:** Sidra Ahsan Shah, Wajeeha Iqbal, Muneeba Sheraz, Bilal Javed, Syeda Sadaf Zehra, Hafiza Aniqa Bint E. Abbas, Waris Hussain, Abdullah Sarwer, Zia-ur-Rehman Mashwani

**Affiliations:** ^1^Allama Iqbal Medical College, Lahore, Punjab, Pakistan; ^2^Department of Internal Medicine, Basic Health Unit Noinwala Tehsil Wazirabad, Gujranwala, Punjab 52000, Pakistan; ^3^Khawaja Muhammad Safdar Medical College, Sialkot, Punjab 51310, Pakistan; ^4^Department of Internal Medicine, Basic Health Unit Ghagga Mitter, Wazirabad, Punjab 52000, Pakistan; ^5^Rawalpindi Medical University, Rawalpindi, Punjab 46000, Pakistan; ^6^Department of Internal Medicine, Basic Health Unit Mitranwali Daska, Sialkot, Punjab 52220, Pakistan; ^7^School of Food Science and Environmental Health, College of Sciences and Health, Technological University Dublin, Dublin, Ireland; ^8^Department of Botany, PMAS Arid Agriculture University, Rawalpindi, Punjab 46300, Pakistan; ^9^Department of Botany, The Islamia University of Bahawalpur, Bahawalpur, Pakistan; ^10^Fatima Jinnah Medical University, Lahore, Punjab 54000, Pakistan; ^11^Nawaz Sharif Medical College, University of Gujrat, Gujrat, Punjab 50700, Pakistan; ^12^Allama Iqbal Memorial Teaching Hospital, Sialkot, Punjab 51310, Pakistan

## Abstract

Bajwat Wildlife Sanctuary is a complex riverine ecosystem and is unique because of the presence of river Chenab, various seasonal streams, lakes, and Head Marala barrage. These ecogeographic conditions provide diverse natural habitats for various plant and animal species to grow uninterrupted and have undocumented ethnopharmacologically important medicinal flora. The present study involves the first-ever extensive investigation to document the ethnopharmacological knowledge on medicinal plants of local healers and inhabitants of the Bajwat Wildlife Sanctuary to treat ailments. The unstructured and semistructured interviews of the local healers and inhabitants were conducted that included 130 individuals. The ethnomedicinal formulations, their method of preparation, mode of administration, parts of the plant used, diseases cured, and their categorization along with species use report (UR) were analyzed. The ethnopharmacological study led to the enlisting of 114 medicinal plant species belonging to 97 genera and distributed among 47 plant families. 2029 URs were collected with 42 general disease categories. Each plant species was reported 18 times to cure various diseases (∼18 UR), while ∼48 URs were collected on each disease category by local informants. Digestive issues (290 URs, ∼14.29%) and skin infections (279 URs, ∼13.75%) were found most commonly among the occupants of the area. The oral administration (69%) of herbal drugs and the preparation of plant extracts (32%) were the most common ethnopharmacological strategies. Inhabitants of the area were well aware of the limited use of poisonous plants. 8 (∼7%) out of the total 114 medicinal plant species were listed in the IUCN Red List of Threatened Species as Least Concern, while *Eucalyptus camaldulensis* Dehnh. was enlisted as near-threatened. The results of the present investigation show that the occupants of the Bajwat have sound information about the ethnopharmacological consumption of medicinal plants, and some of the novel ethnomedicinal formulations were reported which provide the basic data for further pharmacological research.

## 1. Introduction

The traditional herbal medicine system in Pakistan is originated from Ayurveda medicine which has a history of 2500–600 BC [1]. The first documented record of the use of plant medicine in the subcontinent (Indo-Pak) is available in Rigveda (Rigveda is the oldest religious book of the Hindu religion. Many herbal remedies are documented in this book to treat ailments.) and dates to 4500–1600 BC. The herbal medicine system in Pakistan is greatly influenced by the traditional Chinese medicine system, Persian medicines, Greek medicine system [2], and prescriptions from the Prophet Muhammad (PBUH). The *Tib- Al-Nabwi* or Prophetic Medicine system has 1500-year-old history [3, 4]. These diverse features of the traditional healthcare system of Pakistan embellish it with great potential to use plants to treat various ailments.

The tertiary healthcare system in Pakistan is responsible to provide basic to advanced healthcare facilities to the inhabitants. The rural areas in Pakistan have limited healthcare services. Rural healthcare communities have facilities in the form of Rural Health Centers (RHCs) and Basic Health Units (BHUs) that contribute to cover a population of 25,000 inhabitants and are responsible to provide primary healthcare and referral services [5, 6]. Most of the rural communities of Pakistan use herbal medicines because of the limited access to primary healthcare services, expensive medicines, and diagnostic tests [7]. Pakistan is blessed with a great number of higher plants (5,700). Out of the enlisted higher plants, 600–700 are enumerated as therapeutic plants utilized by around registered herbalists and homeopaths. The pharmacopeia endorsed by the National Council of Tibb (Herbalist committee) enlisted 900 medicinal plants commonly used in Pakistan to prepare herbal medicines [8, 9].

Bajwat is situated in the district Sialkot (32°62 N and 74°60 E) and on the outskirts of the district Narowal region of Punjab territory in Pakistan (Figure 1). It contains 84 towns or small villages, with a population of 60,000 as indicated by the 2017 survey. The territory is a wetland of universal significance because of the nearness of Marala Headworks (barrage), Munawar Tawi (river), Jammu Tawi (river), and numerous natural streams, lakes, and muddy regions. Bajwat is situated in a transitional zone between the slopes of Jammu in Indian-occupied Kashmir and the plain zone of Punjab. Bajwat Wildlife Sanctuary has an absolute region of 5,464 hectares which provides free space to wildlife flora and fauna [10]. The most common and universally rare vertebrates of the area include the wild pig or wild boar (*Sus scrofa* L.), deer (*Odocoileus virginianus* Zimmermann), and nilgai (*Boselaphus tragocamelus* Pallas) (blue bull, largest Asian antelope) [11]. These special ecogeographic attributes and the presence of important plant and animal species and serious threats to them contributed to getting the special status for the area [12]. The vast floristic wealth and the rich knowledge of the inhabitants of Bajwat require necessary steps to document this traditional ethnopharmacological knowledge which can help forest officials, NGOs, policymakers, local healers, and researchers that are involved in ethnopharmacological research on medicinal plants. There are very few ethnobotanical studies on medicinal plants reported previously from the district Sialkot [13–17]. These studies were performed superficially, do not provide detailed ethnomedicinal knowledge of the district Sialkot, and do not cover Bajwat Wildlife Sanctuary. The importance of the ethnopharmacological consumption of the medicinal plants of Bajwat Wildlife Sanctuary was ignored, and there was no study to document the significance of the conserved flora.

It was hypothesized that the long-term and well-driven ethnopharmacological survey on medicinal plants of Bajwat Wildlife Sanctuary may help us to enlist ethnopharmacologically important medicinal plants of the area. It can be the first-ever study to document the ethnopharmacological knowledge of the local inhabitants and healers to use plants to treat diseases.

### 1.1. Aim of the Study

The present study was aimed to significantly establish the first-ever inventory of therapeutically important medicinal plants of the Bajwat Wildlife Sanctuary, which is endowed with unique biodiversity and gained a special status to conserve the local flora and fauna. The main objective of this study involves the enlisting of therapeutically significant plant species, their medicinal properties, and methods of preparation of the herbal formulations used by the inhabitants of Bajwat to treat ailments. A bibliographical comparison of the floral diversity of the studied area with the previously published scientific literature from the district Sialkot and with the Herbal Pharmacopeia of Pakistan was performed to determine if the species were reported earlier with similar ethnomedicinal preparations at a regional or national level or if it is reported for the first time in this context.

## 2. Materials and Methods

### 2.1. Study Area and Climate

Bajwat is a small village that is located in the district Sialkot, province of Punjab, Pakistan. Sialkot highlights a humid subtropical atmosphere according to the Köppen–Geiger atmosphere classification, with four seasons [18]. The postmonsoon (rainfall season) season from mid-September to mid-November stays hot during the daytime, yet the evenings are cooler with low humidity. In the winter from mid-November to March, days are moderate to cold, with once-in-a-while substantial rainfall. The temperature in winter may drop to 0°C, yet maximum is rarely under 15°C [11]. The precipitation in the region is very high, which sometimes results in flooding and washing of economically important crops. The normal precipitation is 965 mm [12].

The main source of income for the general population is the cultivation of crop plants such as wheat and rice. They also raise livestock for dairy and profit. The people of the Bajwat have their ethnic linkage with the Kashmir province, and the majority of inhabitants are Muslims by religion. Bajwat Wildlife Area was declared as a sanctuary in 1964 by the Government of Pakistan to protect deer, wild pig, and nilgai from hunting and to prevent other serious threats to the flora. The Bajwat Wildlife Sanctuary is enlisted by the IUCN as a classification IV area, which incorporates a complex of common riverine living spaces, close to the Sialkot along the Chenab River and two of its tributaries, reaching out up to the Indian outskirts (Figure 2). The area is usually inaccessible for a large population and is abandoned due to escalated tensions in the adjacent countries as the east side of the area moves along the Indian border [10]. The main realized danger is the unlawful chasing or hunting of animals, for which the zone has been announced as a Game Reserve and is protected by the Wildlife Department of the Government of Punjab, Pakistan. Below Bajwat is a place where the Chenab (river), Jammu (Occupied Kashmir, India), Tavvi (river), and Manavar Tavvi (river) meet at one spot. The Marala Headworks is situated in Bajwat's southwest corner, is a reservoir of the Chenab river water, and contributes to divert water in different territories of adjacent areas to irrigate field crops. The territory between these two channels is being created as the Marala Barrage Park [11]. These special ecogeographic attributes along with our interest led us to choose this region for our study.

### 2.2. Selection of Informants

The informants who had ethnopharmacological knowledge of medicinal plants and used crude formulations in the past or using in routine to treat ailments were selected [19].

### 2.3. Ethnopharmacological Survey on Medicinal Plants and Data Collection

Open meetings were arranged, in which the individuals were met through casual discussion. Every member was interviewed separately, and the data were recorded with great care. The point of open meetings was to evoke people to talk openly, without any stress or anxiety and to collect information about the medicinal attributes of plants that they utilize or have utilized previously. The second step was semiorganized meetings to acquire detailed quantitative and qualitative data and to obtain a wide range of knowledge on explicit issues. The routine activities of the people of Bajwat Wildlife Sanctuary were observed during the study. A composed questionnaire was designed to collect data containing the name, sex, age, and address. In addition, the level of education of the interviewees and the spot and date of the meeting was recorded. The conversation with the interviewees was in Urdu and Punjabi languages. The questionnaires were filled by the researchers. The ethnopharmacological information consisting of the ethnomedicinal properties of the plant, the vernacular name, the plant parts utilized to prepare medicines, plant occurrence, credited therapeutic properties, and the techniques for preparing ethnopharmacological formulations was recorded [20, 21].

### 2.4. Collection of Plant Samples and Their Identification

The plant samples were collected from the Bajwat Wildlife Sanctuary with the help of local healers, herbalists, sellers, and informants. The study area was surveyed from January to the end of November 2019. The plants were identified by the author Waris Hussain with the help of the Flora of Pakistan. The herbarium sheets containing plant specimens were deposited in the herbarium of the Botany Department of PMAS-Arid Agriculture University, and accession numbers were allotted for future reference [22]. The correct and approved botanical names were enlisted throughout this study after verification from the Pakistan Plant Database (e-Flora of Pakistan) (https://www.tropicos.org/Project/Pakistan) and Plant List (http://www.theplantlist.org/).

### 2.5. Quantitative Data Analysis

The data collected from Bajwat was loaded on the Microsoft Office^®^ program MS Excel^®^ spreadsheet. The graphs were plotted, and the data were evaluated in the form of percentages and proportions. The species use reports (URs) per herbal formulation were also recorded, and the greater number of informants per herbal formulation was considered as an indicator of excessive use of that plant in crude drug preparations. The use reports are defined as the number of informants per herbal formulation or ethnopharmacological preparation [21, 23, 24]. Information was considered coherent when it was reported by two individuals at different times. The diseases reported from the Bajwat Wildlife Sanctuary were arranged according to the international disease categories (ICPC-2, International Classification of Primary Care) by WHO (https://www.who.int/classifications/icd/adaptations/icpc2/en/). Reported 114 medicinal plant species were searched in the IUCN Red List of Threatened Species (https://www.iucnredlist.org/) to determine their conservation status.

## 3. Results and Discussion

Bajwat Wildlife Sanctuary is a protected area that allows a great number of plant and animal species to proliferate freely without any human intervention. The studied area is a complex of different riverine and terrestrial territories that provide a great diversity of ecosystems and environmental conditions for the growth and reproduction of various varieties of plant species. To achieve the study goals and to test the hypothesis, 130 individuals, including 80 male and 50 female participants were interviewed. The local respondents belonged to different age groups ranging from 20–71/above. They had different levels of education from primary to university, while 15% of the informants were enlisted as illiterate (Table 1). The seventh author was originally from one of the villages of Bajwat (Pul-Bajwan). He and his family helped greatly to meet local inhabitants and some known healers of the area. The plant vernacular names are also enlisted in Table 2. The vernacular names were similar in both Urdu and Punjabi languages, and it was not possible to differentiate them based on the language. Ten male herbalists (registered with the National Council of Tibb, Pakistan) were also reported from the studied area. It was observed that the male informants were having more detailed knowledge about the plants' local names, their identification, and collection, while the female participants were having significant information regarding the method of preparation of herbal formulations, and their mode of administration.

### 3.1. Medicinal Plants Diversity in Bajwat Wildlife Sanctuary

The ethnopharmacological survey on medicinal plants of the Bajwat Wildlife Sanctuary led to the collection of 47 plant families and 114 medicinal plant species disseminated among 97 genera (Table 2). The distribution of the plant families to be used in ethnopharmacological medicines among the inhabitants of Bajwat Wildlife Sanctuary can be consulted in Figure 3. 10% of the total reported medicinal plant species belong to the family Leguminosae/Fabaceae. Poaceae and Solanaceae occupied the 2^nd^ rank (7%) in the context of the widely exploited medicinal plant species in the Bajwat Wildlife Sanctuary followed by Moraceae (6%), Asteraceae (5%), Apiaceae, Brassicaceae, Cucurbitaceae, Lamiaceae, and Rosaceae (4% each). Caesalpiniaceae was found to be 3% among the reported species. Fabaceae, Poaceae, Solanaceae, and Moraceae account for 30% of the total reported medicinal plant species of the area. The rest of the families were counted as 2%/<2% separately. A similar trend of utilization of medicinal plant families was reported (Farrukh Nisar et al., 2011; Zereen et al., 2013; Rashid et al., 2014) from the flora of Sialkot unlikely the Pakistan Plant Database (Flora of Pakistan) shows Asteraceae as the largest medicinal plant family countrywide (https://www.tropicos.org/Project/Pakistan).

The lifeforms provide great diversity and physiognomic contrast to the ecological habitat. The most common life forms (Figure 4) are reported in the ascending order for the preparation of herbal medicines such as herbs, shrubs, and trees. Some previous ethnobotanical studies on medicinal plants of the district Sialkot also reported herbs as the extensively utilized plant species to treat ailments of the local inhabitants [13, 14, 16, 17].

### 3.2. The Traditional Source of Knowledge and Bibliographic Comparison

The inhabitants of the Bajwat have sound traditional ethnopharmacological knowledge of medicinal plants because of the ancestral strong linkages among nearby individuals and families. The individuals acquire traditional knowledge from the seniors of the clans and keep on transferring it from one generation to another generation. Along these lines, nearby individuals gather therapeutic plants and treat themselves at home. Most of the senior people of the family, who practice medicine, help and guide their other family members and neighboring communities in the treatment of ailments. Both the male and female members of the society were playing a promising role in the transmission of ethnopharmacological knowledge to their next generation. The females used to guide their daughters and their daughters-in-law about the method of preparation of ethnopharmacological preparation and their mode of administration, while the male family members were going with their young kids to collect plants.

The traditional healers revealed from the studied area were having sound information on ethnopharmacologically significant medicinal plants, their method of preparation of formulations, and their mode of administration. The bibliographic comparison with the existing data from the district Sialkot led to the enlisting of 85 new medicinal plant species with novel herbal formulations not reported previously in the published scientific literature which makes ∼75% of the total collected medicinal plant species (Table 2). The ethnopharmacological comparison of the herbal formulations reported from the Bajwat Wildlife Sanctuary with the Pakistan Herbal Pharmacopeia [8] reported 24 new herbal remedies that make 21% of the total enlisted herbal formulations. The species with similar herbal formulations in different ethnomedicinal studies from the district Sialkot are enlisted in the last column of Table 2.

### 3.3. Plant Parts Used in Herbal Therapy

The different plant parts have different properties which help them to treat therapeutic ailments and likewise have significance in crude herbal formulations. 59% of the plants reported from the studied area were edible medicinal plants which show that these plants can be consumed in different forms to treat ailments, e.g., oral intake of drugs and food supplements to treat malnutrition, etc. while 41% of the medicinal plant species were not edible (Figure 5(a)). It shows that most of the plants of the studied area have their utility as food along with their medicinal applications.  Figure 5(b) shows that 51% of reported plant species have their only use in herbal medications while 21% of plants were used as a source of timber followed by 14% of ornamentals in addition to their other medicinal properties. 8% of the plants were utilized as animals' medicine. Most of the animal medicines were given as fodder to treat animals' digestive issues. Some plants were given to animals as a food supplement while some plants were reported effective to eradicate malnutrition. A herbal formulation was prepared from *Argemone mexicana* L. root extract and applied topically to treat animals' skin issues. 6% of the plants of the studied area were exploited as a source of dietary fiber to treat digestive ailments.

The leaves, roots, wood or bark, flowers, herbaceous stem, fruit, and latex were found useful in a multitude of ethnopharmacological drugs, while some herbal formulations involved the use of whole plant material.  Figure 5(c) shows that leaves and fruits play a significant role to make herbal remedies and stand out 19% separately from both categories which make 38% in total. The great proportion of leaves and fruits in herbal formulations show their significance because of the presence of various phytochemicals that are present in these plant parts, while another reason is the ease of availability of these parts. Wood or bark (12%), latex (10%), and flowers (10%) were reported likewise followed by roots (7%) and herbaceous stems (7%). 11% of the formulations reported the use of the whole plant body, while 5% reported the use of plants as a source of dietary fibers. Some formulations also reported the use of rhizomes or bulbs for the preparation of medicines. Some studies on the ethnomedicinal flora of Sialkot also reported the use of different plant parts in various herbal medicines dominated using leaves, fruits, and herbaceous stems, which is in favor of our study [13, 14, 16, 17].

### 3.4. Preparation of Ethnopharmacological Formulations

Preparation of crude plant formulations involves the use of potential phytometabolites to treat ailments. The potency of a herbal drug to cure disease depends greatly on the method of preparation that in actual is the manipulation of the phyto-secondary metabolites to transfer their full potential from the plant part to the perilous part of the body. Table 2 reports the use of medicinal plants in crude herbal formulations against various pathophysiological conditions. This ethnopharmacological survey reported (Figure 6) the use of plant extracts (32%) as a major method for the preparation of herbal drugs, while 11% of the herbal formulations were prepared in the form of decoctions. Some of the herbal remedies were used in the form of food (10%), oil (10%), and fresh plant materials (6%), while other herbal formulations involved cooking (5%) in the the form of food. The preparation of the ethnopharmacological formulations by the inhabitants of the studied area shows that the food medicinal portion is essential to treat the ailments. The people of Bajwat reported that the consumption of crude herbal drugs as food plays a significant role to treat ailments. The inhabitants of Bajwat were adding crude herbal formulations in their routine food and sometimes were preparing special formulations separately to treat ailments. Some of the inhabitants reported the inhalation of smoke (2%) of wood or other plant material to treat respiratory disorders such as bronchitis, cough, and asthma. A similar number (2%) of plant materials were used for the preparation of tincture. 8% of the total reported plant species were used in animal medicine because of their medicinal importance. Some of the plant species were given to animals as fodder to treat digestive disorders of livestock, to eradicate malnutrition, and used as a food supplement. Few herbal medicines were prepared and applied to animals' skin to cure dermal issues. There is no study reported previously from district Sialkot to determine the mode of preparation of herbal formulations by local inhabitants. Our results are contrary to some previously performed work from different territories of Pakistan that reported powder [25] as the best method for the preparation of herbal formulations because of fewer contamination chances of the powder and easy to preserve and reuse. The people of the Bajwat Wildlife Sanctuary claimed that the preparation of the extract is the most feasible and quick strategy that involves the simple method to prepare formulations and its consumption as fresh can increase the efficacy of a drug in case of any severe ailment.

### 3.5. Administration of the Ethnopharmacological Drugs

Some of the inhabitants of Bajwat were well aware of the mode of administration and its significance. According to inhabitants, the mode of administration helps to deliver the drug efficiently and timely to the suffering part of the body.  Figure 7 encodes various modes of administration of herbal formulations reported by the local inhabitants and healers. The oral route stands up with 69% of the total formulations reported. The oral route reported the ingestion of the fresh plant material powder, using teas, tinctures, or decoctions prepared from different plant parts. People of Bajwat also used oils as a laxative to cure digestive disorders, or sometimes different oils were taken orally to enhance vitality and to reduce feebleness and promote vigor. The oral intake of oil from some plant species was also reported as an aphrodisiac (e.g., *Phoenix dactylifera* L.). The second most common mode of administration was reported as the topical application (15%) of the plant crude drug. The topical administration of the plant material in the form of paste prepared from different plant parts was most common among the inhabitants of Bajwat to treat skin disorders such as acne, skin microbial infections, ringworms, and eczema and to treat burn marks. The topical administration also involved the cosmetic enhancement of the skin glow that includes the use of the paste of *Aloe vera*, *Mentha arvensis* aqueous extract spray, and *Azadirachta indica* paste to cure acne and other skin ailments. The cataplasm makes 7% of the total reported plant species from the study area that involves the maceration of different plant parts such as root, stem, and leaves and applied on the skin to treat different types of skin wounds and different degrees of burns and disorders. The cataplasm was also reported to play a futile role to act as an antidote against the stings of snakes, insects, and other organisms. The ointments also contribute to 7% of the reported mode of administration. Most of the ointments were extracted in the form of oils and massaged on the skin surface to cure joint pain and to promote strength among bones and muscles. Very few of the plant materials were smoked (2%) to cure various respiratory disorders such as asthma, cough, bronchitis, and emphysema. Some of the plant parts such as leaves and flowers were smoked as a narcotic and for recreation such as *Nicotiana tabacum*, while some were used as tranquilizers and sedatives. The oral administration was reported extensively in Pakistan Herbal Pharmacopeia as the major mode of administration of herbal formulations [8]. Some studies performed in the nearby territories of Pakistan [26, 27] also reported oral administration as the most common method of administration of herbal drugs.

### 3.6. Diseases and Pathological Conditions

The digestive disorders were reported most common ailments of the inhabitants of Bajwat which account for 21% of the total disorders cured (Figure 8). Commonly reported digestive disorders include diarrhea, stomach pain, heart-burning issues, nausea, constipation, abdominal bloating, dyspepsia, and vomiting. Different ailments were categorized according to the WHO International Classification of Primary Care, 2^nd^ Edition, which is used worldwide. Skin disorders were found common among the inhabitants to be treated by crude formulations, and 16% of the total ailments cured marked to this category. The most common skin ailments among the inhabitants of Bajwat were reported to be eczema, skin boils, acne, skin burns, skin infections, ringworm, and warts. 14% of respiratory disorders were cured such as cough, asthma, bronchitis, emphysema, and shortness of breath. The rest of the different ailments including fever and malaria (12%), urinary disorders (10%), hepatic ailments (9%), reproductive disorders (7%), cardiac disorders (6%), and neurological disorders (5%) were cured by using different herbal formulations.

Table 3 shows that a total of 2029 URs were collected from 130 informants against 42 pathophysiological groups by using 114 medicinal plant species, and on average, 48 URs were collected against each disease category. Each medicinal plant species was mentioned ∼18 times to cure the health issues of the local inhabitants (∼18 UR per plant species). 290 URs (∼15%) were reported from 32 plant species to treat digestive disorders which shows that digestive disorders are the most common ailments prevailing among the inhabitants of the Bajwat Wildlife Sanctuary, while 279 URs (∼14%) from 27 plant species were mentioned that involved the preparation of different extracts, ointments, and paste for oral and topical administrations to treat skin disorders. There was no study performed previously to report the health disorders of the people of the district Sialkot or inhabitants of the Bajwat Wildlife Sanctuary.

### 3.7. Side Effects of Poisonous Medicinal Plants

The inhabitants of Bajwat reported that most of the plants of the sanctuary do not have any harmful effects. A few species anyway were having dangerous impacts and the nearby individuals keep up broad information about the distinctive poisonous and nonharmful medicinal plants. For instance, the juice of the seeds of *Datura innoxia* Mill. [28], *Datura metel L*. [29], and *Ricinus communis L*. [30] is known to be profoundly harmful. A few plants were reported to have poisonous impacts on both humans and livestock, for example, *Calotropis procera* (Ait.) and *Euphorbia helioscopia L*. The latex of the two plants causes harmful impacts through eye and skin contact. Some studies reported that the use of the limited dose of the latex of *Euphorbia* is beneficial to treat warts and wounds, but excessive and unlimited use of latex can be carcinogenic [21]. *Parthenium hysterophorus* L. was also reported to be a poisonous plant by local healers and some inhabitants and can cause severe respiratory ailments and was found growing excessively along the roadsides. Although some people in the local market were found using *Parthenium hysterophorus* L. to decorate flower bouquets, Maleki and Akhani [21] also reported some of the plants mentioned above as poisonous plants from Mountain Taftan, Iran, which is located at the border of Pakistan's southwestern province, Balochistan. The Royal Botanical Garden's annual report [31], stated 8% of poisonous plants out of the total documented plant uses. However, in the Bajwat Wildlife Sanctuary only 6 plants were reported poisonous which makes 5.26% of the total reported plant species of the study area.

### 3.8. Plants Enlisted in the IUCN Red List of Threatened Plant Species

The IUCN Red List of Threatened Species provides significant information about the evidence-based extinction and risk assessments of individual plant species. It also contributes to understanding the forces that are responsible for the extinction of species and also helps in management interventions to overcome or delay the extinction. Despite critical evaluation of species at risk of extinction, it is believed that many plant species will be extinct before they have been recognized as being at risk of extinction [32]. Determination of plant species' current status in the IUCN Red List of Threatened Species can greatly help to protect the threatened ethnomedicinal flora of a region. According to the IUCN Red List of Threatened Plant Species, more than 3200 species are threatened with extinction, which makes about 27% of the total assessed species. Eight out of the total 114 plant species were listed in the IUCN Red List as least concern (LC), including *Bauhinia variegate∗*, *Cyperus rotundus* L., *Cassia fistula* L.*∗*, *Centella asiatica* (L.) Urb.*∗*, *Echinochloa crus-galli* (L.) P. Beauv, *Eclipta prostrata* L., *Vitis vinifera* L.*∗*, and *Vitex negundo* L. while *Eucalyptus camaldulensis* Dehnh.*∗* was enlisted as near-threatened (NT). The occurrence of plant species in Bajwat Wildlife Sanctuary was also observed, and 19 species were found rarely distributed, which makes 17% of the total reported plant species, while 5 species (*∗* placed at the end of their name) out of 19 rarely distributed species were enlisted in the IUCN Red List of Threatened Species (Table 2).

## 4. Conclusion

This study involves the first-ever extensive ethnopharmacological investigation to report the medicinal plants of the Bajwat Wildlife Sanctuary, which is a complex riverine biological ecosystem. We have reported 114 medicinal plant species. The extract preparation (32%) was reported as the most basic strategy for making herbal formulations, while oral intake (69%) was observed most common for the administration of drugs among the local community. The highest number of URs against digestive disorders (290∼15%) and skin disorders (279∼14%) show that these are the most common problems among the local inhabitants. The stomach-related issues were seen generally regular among local people and were cured by crude ethnopharmacological formulations. This study embraces the ethnopharmacological knowledge of local healers and inhabitants and reports the exchange of data from generation to generation because of strong communication in families and neighboring communities. The investigation of the ethnomedicinal information and their comparison with past reports from the district Sialkot, and Pakistan Herbal Pharmacopeia endorses the enlisted knowledge of local healers and inhabitants to prepare formulations against multiple disease categories. About 75% of the enlisted medicinal plant species were not reported previously in research reports from Sialkot, while 21% of novel herbal formulations were documented in comparison with the Pakistan Herbal Pharmacopeia. This study likewise explains the importance of the studied zone and the incredibly assorted diversity of plants and its status to help plant species to develop unreservedly without human mediation.

## Figures and Tables

**Figure 1:** The map of Pakistan showing its neighboring countries and the site of the study. The south of Pakistan is lined by the Arabian coast. The red highlighted map shows the location of Sialkot and the green dot represents the location of the Bajwat Wildlife Sanctuary.

**Figure 2:** The photographic images of different areas of the Bajwat Wildlife Sanctuary. (a) Bridge on the river Tawi and the grassland; (b) the forest is flooded with water during monsoon season after heavy rainfall; (c) the inhabitant is using an animal cart to carry plants; (d) waterways in the study area; (e) plants growing freely in the protected area; (f) Head-Marala barrage.

**Figure 3:** The percentage distribution of medicinal plant families among Bajwat Wildlife Sanctuary. 47 families disseminated among 97 genera and 114 medicinal plant species represent the great diversity of plants.

**Figure 4:** The life form of different plant species.

**Figure 5:** (a) The percentage distribution of the edible and nonedible plants. (b) The percentage distribution of the modes of the plant used. (c) The distribution of different parts of plants for making herbal formulation.

**Figure 6:** The diagram represents the method of preparation of crude ethnopharmacological drugs.

**Figure 7:** The diagram represents the mode of administration of crude plant drugs.

**Figure 8:** The diagram showing the percentage of different disorders cured by using plant formulations.

**Table 1:** Statistic and Socio-cultural factors of Interviewees.

Factors	Items	Numbers (♂ + ♀)	Percentage
Gender	Male	80	61.53
	Female	50	38.46

Age groups	20–30	23 + 7	23.07
	31–40	27 + 8	26.92
	41–50	12 + 13	19.23
	51–60	10 + 10	15.38
	61–70	6 + 9	11.53
	71 and above	2 + 3	3.84

Herbalist	Male	10	7.69

Educational level	Illiterate	12 + 8	15.38
	Primary	20 + 15	26.92
	Middle	5 + 5	7.69
	High school	12 + 8	15.38
	Higher secondary	20 + 10	23.07
	University	7 + 3	7.69
	Others	4 + 1	3.84

♂ represents male participants, and ♀ represents female participants.

**Table 2:** List of plants with voucher numbers, their families, vernaculars written in English and Urdu, different plant parts to treat ailments, mode of administration, life forms, occurrence, and use reports (URs) for each preparation and their reported ethnomedical uses.

Family/species (accession no.)	Vernacular (Urdu name)	Part(s) used	Disease(s) treated/other uses	Mode of preparation(s) (UR against each disease)	Mode of adm.	Life form	Occurrence	Similar use(s) references
Adiantaceae/*Adiantum philippense* L. (BWS-066)	Chota kalbatra (چھوٹا کل بترا)	Leaves, rhizome	Infections, fever/blood purifier	The decoction of the rhizome is used to treat fever and febrile conditions in children (2). Plant extract is used as a blood purifier (2). The juice is applied to skin infections (1).	Oral, topical	HB	Rare	
Alliaceae/*Allium cepa* L. (BWS-069)	Piaz, ganda (پیاز ,گنڈا)	Leaves, bulb	Dyspepsia, stomach issues, inflation, diabetes/antiseptic, sting treatment	Macerated infusions and juice are used for the treatment of dyspepsia (17), stomach pain (12) and acute catarrhal inflation (10). Macerations are used against snake bites and other stings (15).	Oral, cataplasm	HB	Common	*∗*
*Allium sativum* L. (BWS-068)	Thom (تھوم)	Leaves, rhizome	Diabetes, cholesterol, skin infections, bites of insects, spiders and snakes, hypertension, kidney stones	Used as a condiment and for treatment of dyspepsia (7) and the constant rattling of mucus in bronchi (11). Extract and maceration are used on skin infections and bites (12). Chewing cloves helps to manage hypertension (15). The juice is used for kidney stones (12).	Oral, cataplasm	HB	Common	*∗*
Amaranthaceae/*Achyranthes aspera* L. (BWS-067)	Putthkanda (پوٹھکنڈا)	Whole plant	Blindness, cough, asthma treatment, scorpion bites, kidney stones/antilithic, analgesic	Decoctions are prepared with other medicinal plants used for cough (2) and to relieve pain (1). Leaves are used for UTIs treatment (4). The whole plant is used for kidney stones (3). Extracts are used for eye infections (1).	Oral, eye drops, topical	HWB	Common	[13]*∗*
*Amaranthus spinosus* L. (BWS-070)		Whole plant	Leucorrhoea, habitual abortion, vomiting, allergic asthma, fever, piles and leprosy	Tinctures and decoctions are used for the mentioned diseases. Decoctions are used to induce abortion (1), vomiting (1), fever (2), piles (1), and leprosy (1).	Oral	HWB	Common	
Anacardiaceae/*Mangifera indica* L. (BWS-072)	Aamb (آم)	Whole plant	Scorpion stings/digestive issues treatment, blood purification, induce child delivery	The leaf extract is applied to scorpion-sting (4). Decoctions are used for digestive issues (6). Fruit induces delivery (2) and juice as a blood purifier (3).	Oral, topical	TT	Common	*∗*
Apiaceae/*∗Centella asiatica* (L.) *Urban* (BWS-071)	Ghhor sumbi (گھوڑ سمبی)	Whole plant	Brain health, digestive disorders	Brain tonic (1), plant tablets are a strong drug for mentally retarded children (3). The plant extract is used for digestive disorder treatment (3).	Oral	CP	Rare	
*Coriandrum sativum* L. (BWS-062)	Dhannia (دھنیا)	Seeds, oil, leaves	Carminative, bile issues and hypertension treatment, skin treatment	Extract and decoctions are used. Dilute aqueous extracts are used as a cooling agent to treat hypertension (10). Leaves extracts and teas are used for digestive disorders (15). Oils and extracts are used to treat dry scalp (10). The seed extract is antibacterial and sedative used in lotions and shampoo (15).	Oral, ointments, cataplasm	GH	Common	*∗*
*Carum copticum* L. (BWS-063)	Daisi ajwain (دیسی اجاوین)	Seeds	Stomach trouble, fever, malaria, and flu	Oil is extracted, used for flu (7). Decoctions and the powder are used for stomach treatments (6). Seeds are used as masticatory (7). Leaves and seeds are used for malaria and fever (5).	Oral, ointment	GH	Common	*∗*
*Daucus carota* L. (BWS-065)	Gajar (گاجر)	Roots, seeds	Improve vision, blood purification, anemia treatment	Extracts are prepared and used for the treatment of anemia (20) and the purification of blood (10). Juice and extract are used to improve vision (30).	Oral	HB	Common	*∗*
*Foeniculum vulgare* Mill. (BWS-064)	Saunf (سونف)	Seed, oil, leaves	Infections, fever, liver issues, digestive issues/blood purification	Leaves and seed extract are used in fever (12), liver (2) and digestive complaints (8), seeds cooked in milk increase lactation and nourishment (12). Oil from seeds is vermicide and antimicrobial (12).	Oral	HB	Common	*∗*
Apocynaceae/*Nerium indicum* Mill. (BWS-073)	Kanera (کنیرا)	Roots, leaves	Promotes abortion	The root powder is used for the preparation of drugs to promote abortion (5)	Oral, ornamental	SH	Rare	*∗*
*Catharanthus roseus* (L.) G. Don (BWS-074)	Sadaa bahar (صدا بہار)	Leaves	Digestive disorders	Leaves extracts and decoctions are prepared to relieve constipation (4) and digestive issues (4)	Oral, ornamental	HB	Common	[17]*∗*
Arecaceae/*Phoenix dactylifera* L. (BWS-059)	Khajoor (کھجور)	Leaves, fruit	Aphrodisiacs, hepatic treatment, anemia treatment	Edible fruit, rich in sugar, useful tonic (7). Fruit boiled with goat and cow milk is used as an aphrodisiac (10). Fruit helps to treat anemic conditions (8).	Oral	MP	Rare	[17] *∗*
Asclepdiaceae/^**†**^*Calotropis procera* (ait.) ait. f. (BWS-060)	Ak sinn (اک سن)	Leaves, roots, flower	Infections, pneumonia, leprosy/antidote	Young leaves together with onion and salt are used in snakebite (12). Milky juice cures skin infections (8). Latex is used for the treatment of pneumonia fever (2) and leprosy (2). Poisonous plant.	Oral, cataplasm	SB	Common	[17]*∗*
Asteraceae/*Ageratum conyzoides* L. (BWS-001)		Whole plant	Asthma, bronchitis/stops bleeding, postpartum recovery	Plant extract and juice are prepared for asthma (3) and other respiratory disorders and postpartum recovery (5). The paste is used to stop bleeding (3).	Oral, topical	BSH	Common	
*Cichorium intybus* L. (BWS-061)	Kasni (کاسنی)	Roots, leaves	Hepatitis A, B, and C, kidney disorders, digestive disorders	Extract from leaves, used in jaundice (3) and other liver complaints (3) and digestive disorders (2)	Oral	HB	Common	*∗*
*Eclipta alba* (L.) Hassk. (BWS-075)	Bhangra (بھنگڑا)	Whole plant	Skin infections, hepatic ulcers	Plant paste is used for the treatment of skin infections (3). The decoction of the leaf is a liver tonic (2).	Oral	HB	Common	[17]*∗*
^**†**^ *Parthenium hysterophorus* L. (BWS-057)	Kauri booti (کوڑی بوٹی)	Leaves, flowers	Diabetes, cold, fever, poisonous plant	Extracts are used for the treatment of diabetes (7) and fever (2). The plant is poisonous and causes various respiratory tract allergies and infections.	Oral	SB	Common	*∗*
*Tagetes erecta* L. (BWS-056)	Gutta, jangli satt barga (گٹہ ،جنگلی ست برگہ)	Leaves, flowers	Wound, injuries, snake bites, UTIs/antiseptic, hepatoprotective	Extracts, decoction, juice and powder are prepared for the treatment of liver (3), kidney stones (3). The paste is applied to the bites of the snake (2).	Oral, cataplasm, ointment	HB	Common	
*Xanthium strumarium* L. (BWS-058)	Jojra (جوجرا)	Root, leaves, fruit	Smallpox/antimalarial, cancer treatment, improve vision	Decoctions are used in the treatment of long-standing malaria (4). Roots are used to treat cancer (3). The fruit is used in smallpox (2) and eye ailments (3).	Oral, ointments	SB	Rare	[17] *∗*
Bombacaceae/*Bombax ceiba* L. (BWS-076)	Simbal, sumbal (سمبل ،سنبل)	Whole plant and its products	Bleeding gums, toothache and sores in the mouth, enlargement of spleen	Branches are used as a masticatory and toothbrush. Powder and fresh leaves are chewed to relieve bleeding gums (2) and toothaches (2). Decoctions are used to treat enlarged spleen (3).	Oral	TT	Common	[13]*∗*
*Bombax* spp (BWS-034)	Barru ghas (بارو گھاس)	Stem and inflorescence	Digestive disorders	The inflorescence is used to treat digestive disorders (6)	Oral, other	HB	Common	[13]*∗*
Brassicaceae/*Brassica nigra* (L.) Koch (BWS-077)	Saroon (سروں)	Leaves, seeds, oil	Antiseptic, joint pains	Oil is antiseptic (7) and used for joint pain (8)	Oral, ointment	HB	Common	*∗*
*Capsella bursa-pastoris* (L.) Medik. (BWS-079)		Leaves	Uterine infection	Infusion from the plant is prepared to treat uterine infections (5)	Oral	HB	Common	*∗*
*Eruca sativa* Mill. (BWS-010)	Tara mera, kara bara (تارا میرا ،کارا بارا)	Leaves, seeds, oil	Scabies, dandruff/antiseptic, antiallergic, skin treatments	Seeds oil is highly antiseptic (5); used to cure itching (7), and skin infections (7). Oil cake is used as cattle feed to cure digestive ailments (3).	Topical	HB	Common	*∗*
*Raphanus sativus* L. (BWS-081)	Mooli (مولی)	Leaves, roots, flowers, fruit	Stomach pain, ringworm/laxative, digestive treatment, kidney stone treatment	The root is eaten as food. Decoctions cure stomach troubles (9). The water of leaves cures ringworm (8). Pods are used as a vegetable. Root water is extracted to cure kidney stones (10).	Oral	HB	Common	*∗*
Caesalpiniaceae/*Bauhinia racemosa* Lamk. (BWS-080)		Whole plant	Diarrhea, dysentery, ulcers, inflammation, biliousness, UTIs	Root bark extracts are used to treat diarrhea (3), dysentery (2), stomach ulcers (2), kidney stones (2) and inflammation (1). Stem bark extract cures biliousness and urinary discharge (1).	Oral	BT	Rare	
*∗Bauhinia variegata* L. (BWS-078)	Kachnar (کچنار)	Bark, leaves, seed, root, flowers	Ulcers, gastrointestinal disorders, and piles	The extract is used to cure stomach ulcer (4) and digestive disorders and piles (2)	Oral	TR	Rare	*∗*
*∗Cassia fistula* L. (BWS-002)	Amaltas (امالتاس)	Fruit, root bark, stem leaves, flower	Skin disease, heart diseases, stomach ulcers and relieve heartburns, tuberculosis	Topical applications treat skin diseases (2). The root extract is useful in tuberculosis treatment (2) and burning sensation (2). Seeds extracts are emetic (1). Fruit extract cures leprosy (2). Pod tea is used to cure cough (7).	Oral, topical	TR	Rare	[17]∗
Cannabaceae/*Cannabis sativa L*. (BWS-088)	Bhang (بھنگ)	All parts	Narcotic, nervous disorders, e.g., epilepsy, mania, dementia, irritable reflexes	Plant aqueous extracts are prepared separately or with different plants for treatments. Dried leaves are smoked as narcotics (12). Leaves and flowers are smoked to cure nervous disorders (8).	Oral, inhaled	SB	Common	[17]*∗*
Chenopodiaceae/*Chenopodium album L*. (BWS-084)	Bathu (باتھو)	Vegetative parts, seeds, oil	Digestive disorders/insecticidal, hepatoprotective	Flowers and buds are used in stomach troubles (6). Seeds are used in hepatic disorders and spleen enlargement (2). Oil kills worms (1).	Oral	HB	Common	[13]*∗*
*Chenopodium ambrosioides* L. (BWS-087)	Kurund (کرونڈ)	Vegetative parts	Insecticidal	Used to kill insects (3)	Oral	HB	Common	
Convolvulaceae/*Convolvulus arvensis L*. (BWS-085)	Leli (لیلی)	Whole plant	Digestive disorders, respiratory disorders, kidney stones	The whole plant is purgative and extracts are prepared for the treatment of cough (2). Tea is prepared to remove kidney stones (2).	Oral	CP	Rare	[13]*∗*
Crassulaceae/*Kalanchoe pinnata* (lam.) Pers (BWS-086)	Patthar chat (پتھر چٹ)	Leaves	Kidney stones, wound treatment, ringworms, and other skin disorders	Leaves are eaten with common salt to treat kidney stones (5). Juice of leaves is applied to injuries (4) and ringworms (2).	Juice, cataplasm	HB	Rare	*∗*
Cucurbitaceae/*Cucumis melo-var agrestis* Naudin. (BWS-083)	Chibra (چبڑا)	Fruit, seeds	Digestive disorders	Fruit and seeds extracts are used to cure digestive malfunctioning (7)	Oral	CP	Common	[17]*∗*
*Momordica charantia* L. (BWS-082)	Karela (کریلہ)	Fruit	Malaria, skin disorders/dengue treatment, antiseptic	The water of fruit is used as a blood purifier (12) and for dengue (5) treatment. The paste is applied to the skin to treat infections (9).	Oral, topical	CP	Common	*∗*
*Citrullus lanatus* (thunb.) mats. and Nakai (BWS-089)	Tarbooz, dawana (تربوز ،ڈوانا)	Fruit, seeds	Digestive disorders, fever	The fruit is used as a cooling agent (9). Cotyledons of seed are used to cure digestive disorders (3).	Oral	CP	Common	*∗*
*Luffa acutangula* (L.) Roxb (BWS-003)	Kali tori (کالی توری)	Fruit	Digestive disorders/laxative	Extracts are prepared for the treatment of constipation and digestive issues (4)	Oral	CRH	Common	
Cuscutaceae/*Cuscuta reflexa* Roxb. (BWS-090)	Akash bail (آکاش بیل)	All parts	Kidney stones treatment, hepatic disorders	It is purgative and extracts are used in the liver (4) and kidney disorders (3)	Oral	PE	Common	*∗*
Cyperaceae/*∗Cyperus rotundus* L. (BWS-009)	Dela (ڈیلہ)	Rhizome	Digestive disorders, fever, cardiac disorders	The tuber is useful in stomach disorders (1). Soup of tuber is useful in diarrhea, dysentery, dyspepsia, vomiting, cholera (1) and fever (1). Whole plant juice is prepared for heatstroke (1).	Oral	RH	Common	[17]
*Cyperus scariosus* R.Br. (BWS-028)	Bara dela (بڑا ڈیلہ)	Rhizome	Digestive disorders, fever, cholera	The tuber is useful in stomach disorders (1). Soup of tuber is useful in diarrhea (1), dysentery, dyspepsia, vomiting, cholera and fever (1).	Oral	RH	Common	*∗*
Equisetaceae/*Equisetum spp*. (BWS-091)	Baansi booti (بانسی بوٹی)	Whole plant	Cough treatment	Tea is used to treat dry cough (5)	Other	HB	Common	
Euphorbiaceae/**† ***Euphorbia helioscopia* L. (BWS-004)	Daddar booti (دادار بوٹی)	Latex, leaves	Ringworm treatment, narcotic, constipation	The plant is narcotic and a little poisonous. The milky latex is applied to skin infection especially in ringworm disease (4). Extracts are used for digestive disorders (2).	Oral, topical	HB	Common	*∗*
**† ** *Ricinus communis* L. (BWS-006)	Dhola, airn, arind (ڈھولہ ،ایرن ،ارنڈ)	Oil, seed, root	Digestive disorders, joint pains, poisonous plant	Oil and decoctions are used in the treatment of constipation (4), also increase milk production (3) and treatment of painful joints (3). The extract is used for stomach ulcer treatment (6).	Oral, topical	MT	Common	[17]*∗*
Fumariaceae/*Fumaria indica* (hausskn.) Pugsley (BWS-093)	Shahtara (شاہتارا)	Whole plant	Blood purification, sweating treatment	Whole herb extract is used as a blood purifier (6). The extract is prepared to treat excessive sweating (3).	Oral	HB	Common	*∗*
Fabaceae/*Cicer arietinum* L. (BWS-026)	Chana (چنا)	Seeds, leaves	Leucorrhea, animals' medicine	Roasted grams aqueous extracts are said to be beneficial in leucorrhea (10). Seed coats used as a food supplement for livestock.	Oral	SH	Common	*∗*
*Lens culinaris* Medik. (BWS-092)	Massur (مسور)	Seeds	Cold and fever	Seeds are used in the treatment of fever and cold (3)	Other	SH	Common	*∗*
*Pisum sativum* L. (BWS-005)	Matar (مٹر)	Seeds	Food	Green unripe seeds and ripened seeds are used as pulses and vegetable (3)	Other	SH	Common	*∗*
*Melilotus indica* (L.) All. (BWS-011)	Methri (میتھری)	Leaves	Respiratory disorders, digestive ailments	Seed powder is used in asthma treatment (4). Decoctions are recommended into abdominal ailments (3).	Oral	SH	Common	*∗*
*Medicago polymorpha* L. (BWS-094)	Maina (مینا)	Leaves, buds	Infections	Skin infections (5)	Other	SH	Common	*∗*
*Trigonella foenum-graecum* L. (BWS-027)	Methy, methry (میتھی ،میتھرے)	Leaves, seeds	Respiratory disorders, kidney disorders, fever, joint pain	Seeds are used in asthma (2), fever (1), sore throat (2) and pains in the body (2)	Oral	SH	Common	*∗*
*Dalbergia sissoo* Roxb. (BWS-012)	Tahli (تہلی)	Bark and wood	Digestive disorders	Decoctions and juice are prepared from leaves for the treatment of digestive disorders (11)	Oral	TR	Common	[13]*∗*
*Sesbania sesban* (L.) Merrill (BWS-018)	Janter, jantri (جنتر جینتری)	Fiber, wood, seeds	Animals' medicine	The seed is used as a food supplement for livestock (7)	Other	SB	Common	
*Crotalaria juncea* L. (BWS-007)	Sann (سان)	Stem, fiber	Digestive treatment	Fiber is used as a laxative (10)	Other	SB	Common	
*Pongamia pinnata* (L.) Pierre. (BWS-019)	Sukh chan (سکھ چین)	Shoots	Dental issues, skin disorders	Shoots are used to make toothbrushes (11). The paste is used for the treatment of skin disorders such as ringworms (6).	Oral, tropical	TR	Common	[13]*∗*
Lamiaceae/*Leucas aspera* (willd.) Link (BWS-095)	Piddu (پڈو)	Leaves, flowers and fruit	Antimalarial, respiratory disorders	Extract of leaves, flowers and fruit are used as an antimalarial drug (4). The extract is used to treat cough (2).	Oral	SB	Common	[17]*∗*
*Mentha arvensis* L. (BWS-008)	Podina (پودینا)	Leaves, whole plant	Digestive disorders, dermal treatment	Syrup of leaves used in digestive diseases (30). Extracts are used in cosmetic products (24).	Oral, topical	SB	Common	*∗*
*Ocimum basilicum* L. (BWS-013)	Niazbo (نیازبو)	Leaves, seeds	Headache, fever	Tea is prepared from leaves to relieve headaches (12). Extracts have a potential role to treat fever (12).	Oral	HB	Common	*∗*
*Salvia splendens* sellow ex Schult. (BWS-096)	Sinji (سنجی)	Whole plant	Animals' medicine	Used to treat livestock digestive disorders (8)	Other	SH	Common	
Liliaceae/*Aloe vera* (L.) burm. f. (BWS-054)	Kavaar gandal (کوار گندل)	Leaves, pulp	Dermal treatment, joint pains	Leaf pulp is a skin tonic and is used in medicines and cosmetics (25). Pulp cooked in milk is useful in joints pain (35).	Ointment, topical, cataplasm	HB	Common	[17]*∗*
Linaceae/*Linum usitatissimum* L. (BWS-024)	Alsi (السی)	Seeds, fiber	Gout treatment, rheumatic issues, food, laxative, animals' medicine	Seeds are used in rheumatic (10) and gout swellings (2). Laxative in the case of hemorrhoids (11). Oil is edible. Oil cake is a cattle food supplement (2).	Oral, ointment	HB	Common	
Malvaceae/*Abutilon indicum* (L.) Sweet. (BWS-025)	Muhri booti (مہری بوٹی)	Bark, seed, root	Infections, fever, digestive disorders, respiratory and neural issues	Leaf paste applied in fever (4) and headache (4). Flowers are used for boils (1) and stomach ulcers (2). Seeds are used as a laxative (4). Powder of flowers, fruit and root is used in cough (2) and leprosy (1).	Oral, topical	HB	Rare	*∗*
*Hibiscus rosasinensis* L. (BWS-020)	Chini gulab (چین گلاب)	Flower petals	Kidney stones	Extracts are used for the treatment of kidney stones (11)	Oral	SB	Common	[17]*∗*
Meliaceae/*Azadirachta indica* (adr. Juss.) (BWS-014)	Neem (نیم)	Wood, leaves, fruit	Blood purifier, dermal treatment	Leaves are used as skin tonic in cosmetics and skin diseases (40). Extract of leaf purifies the blood (10). The fruit is edible.	Oral, topical, cataplasm	TR	Common	[13]*∗*
*Melia azedarach* L. (BWS-015)	Dharek (دھریک)	Leaves and wood	Blood purifier, infections treatment, dermal disorders, diabetes	Wood and leaf extracts are blood purifier (30), it cures diabetes (20)	Oral, topical, cataplasm	TR	Common	[17]*∗*
Mimosaceae/*Acacia nilotica* (L.) Delile (BWS-055)	Kikri (ککری)	Bark, leaf, fruit	Respiratory disorders, digestive issues	The bark is used to cure cough (12) and dysentery (10). Leaves cure stomach ulcers (5). Pods and seeds are also medicinal.	Oral	MT	Common	[17]*∗*
*Albizia lebbeck* (L.) Benth. (BWS-023)	Sharin (شریں)	Bark, gum, wood	Respiratory ailments, digestive disorders, laxative, relieve pain	Extracts are used for the treatment of various respiratory (5) and digestive ailments (5). Bark and gums are of medicinal values and used as a laxative (6).	Oral	TR	Common	*∗*
Moraceae/*Broussonetia papyrifera* (L.) L'Herit. (BWS-053)	Jangli shehtoot (جنگلی شاہتوت)	Wood	Respiratory ailments	Used to treat respiratory disorders of livestock (10) and humans (7)	Others	TR	Common	*∗*
*Ficus carica* L. (BWS-021)	Angeer, pakwari (انجیر ،پکواری)	Fruit, latex	Wound treatment, digestive disorders, blood purifier	Milk of plant is anti-microbial and is applied to wounds and injuries (10). The fruit is a tonic and cures digestive diseases (16) fruit is available in fresh and dry form, used as a blood purifier (10)	Oral, topical	MT	Common	*∗*
*Ficus palmata* Forssk. (BWS-016)	Jangli pakwari/Anjeer (جنگلی پکواری/انجیر)	Fruit, latex	Wound treatment, digestive disorders	Milk of plant is antimicrobial and is applied to wounds and injuries. The fruit is a tonic and cures digestive diseases.	Oral, topical	MT	Common (19)	
*Ficus glomerata* Roxb. (BWS-017)	Gullar, rumbal (گلر ،رمبل)	Wood, fruit	UTIs treatment, dermal disorders, sexual disorders, digestive disorders	The fruit is used in the treatment of urinary discharges (7), leucorrhea (4), skin diseases (4) and stomach ulcers (5)	Oral	LT	Common	
*Morus acedosa* Griff. (BWS-022)	Shahtoo (شاہتوت)	Fruit, wood	Cough treatment, bronchitis, sputum relieving	Fruit extract and juice are used for respiratory disorders (35)	Oral	TR	Common	
*Morus alba* L. (BWS-032)	Chitta toot (چٹہ توت)	Leaves, fruit, wood	Digestive disorders, hepatic treatment	Edible fruit, laxative (10), increase bile production (10), soothe throat sore (9) and pain in tonsils (10)	Oral	TR	Common	*∗*
*Morus nigra* L. (BWS—029)	Kala toot, toot sia (کالا توت)	Leaves, fruit, wood	Food, digestive disorders, hepatic treatment, respiratory disorders	The syrup is made from fruit which cures cough (13) and sore throat (12). Other uses are the same as in the case of *M. alba*	Oral	TR	Common	[17]*∗*
Myricaceae/*Psidium guajava* L. (BWS-031)	Amrood (امرود)	Fruit	Digestive disorders, respiratory infections	Nutritive fruit, good for digestive tracts (20), medicinal in case of diarrhea (12). Ashes of dried fruit are used for the treatment of whooping cough (20).	Oral	TR	Common	*∗*
Myrtaceae/*∗Eucalyptus camaldulensis* Dehnh (BWS-097)	Safeda (سفیدہ)	Wood, leaves	Cold, cough, fever	Leave extracts and tinctures are used for the treatment of cough (13) and cold (12)	Oral	TR	Rare	
Oleaceae*/Jasminum grandiflorum* L. (BWS-052)	Chambeli (چمبیلی)	Root, leaves, flowers	Dermal issues	The plant is used for healing chronic ulcers (12), skin diseases (12) and poisonous infections. Roots are used for ringworm (12).	Oral, topical	SB	Common	*∗*
*Jasminum sambac* (L.) Ait. (BWS-030)	Motia (موتیا)	Root, leaves, flowers	Dermal disorders, ringworm treatment, digestive disorders, eye disorders	The plant is used for healing chronic stomach ulcers (12), skin diseases (10) and poisonous infections (10). The root is used for ringworm treatment (10). Leaves boiled in oil are used as a balm which is used for anointing the head in eye complaints and to improve vision (12).	Oral, topical	SB	Common	*∗*
Oxalidaceae/*Oxalis corniculata* L. (BWS-101)	Khatti booti (کھٹی بوٹی)	Whole plant	Food, dyspepsia, piles, anemia, fever, dysentery, scurvy	The plant is medicinal, aqueous extracts cure dyspepsia (4), piles (2), anemia (2), fever (2), dysentery (3) and scurvy (2)	Oral	HB	Common	*∗*
Papaveraceae/*Argemone mexicana* L. (BWS-098)	Kandiari (کنڈیاری)	Root, seed, juice and oil	Dermal treatment, hepatic disorders, animals' treatment	Seeds are a source of oil; used as a lubricant (8). Root used in chronic skin diseases (2). Plant juice is used in oedema (2), jaundice (2) and cutaneous infections (2). It is also used for cattle skin diseases (2).	Oral, topical, ointments	HB	Rare	
Poaceae/*Arundo donax* L. (BWS-099)	Narr (ناڑ)	Leaves, stem	Menstrual pain, headache	Extracts are prepared and used to relieve multiple pains (3)	Oral, other	SHS	Common	[14]
*Avena sativa* L. (BWS-100)	Jangli jae, jawi (جنگلی جائی ،جاوی)	Vegetative parts	Cardiac disorders, respiratory disorders	Infusions and decoctions are prepared to treat cardiac ailments (4) and respiratory disorders (4)	Oral	HB	Common	*∗*
*Bambusa arundinacea* (retz.) Willd. (BWS-102)	Bans (بانس)	Stem	Joint pain	Powder from stem nodes is used to treat joint pains (12)	Other	LT	Common	*∗*
*Cynodon dactylon* (L.) Pers. (BWS-033)	Khabbal ghas (کھبل گھاس)	Whole plant, leaves	Hemorrhage, anemia, skin infections	Infusion and decoctions are prepared for skin treatment (10). Tinctures are used for the treatment of anemia (12) and hemorrhage (12).	Oral	HB	Common	*∗*
*∗Echinochloa crus-galli* (L.) P. Beauv (BWS-103)	Swank ghaas (ساوناک گھاس)	Leaves	Skin infection	It is used to treat infections (7)	Other	HB	Common	
*Triticum aestivum* L. (BWS-050)	Kanak, gandum (کنک ،گندم)	Straw, seeds	Antiseptic	Extracts are antiseptic (15)	Oral	CLH	Common	*∗*
*Saccharum officinarum* L. (BWS-035)	Ganna (گنا)	Stem	Food, hepatoprotective	Source of sugar. The juice is used to treat jaundice and hepatitis (16).	Oral	CLH	Common	*∗*
*Pennisetum glaucum* (L.) R.Br. (BWS-051)	Bajra (باجرہ)	Whole plant	Malnutrition, weight loss	Extracts are used for malnutrition and weight loss treatment (9)	Oral	CLH	Common	*∗*
Polygonaceae/*Rumex dentatus* L. (BWS-104)	Jangli palak (جنگلی پالک)	Root and vegetative parts	Respiratory disorders, abortifacient	Used as a cough remedy (11). Leaves extracts are prepared to induce abortion (4).	Oral	HB	Common	*∗*
Primulaceae/*Anagallis arvensis* L. (BWS-107)	Kokoo ghass (کوکو گھاس)	Leaves, seeds	Skin disorders, wound healing	Decoctions are used for hydrophobia and dropsy treatment (8). It also cures warts and itching (8).	Topical	HB	Common	
Pteridaceae/*Pteris spp.* (BWS-105)	Kalbatra (کلبترا)	Rachis	Nutrient balance, fertilizer	Help to balance nutrients in the body. It increases Cu++ and As++ ions in soil (5).	Other	HB	Rare	*∗*
Rhamnaceae/*Ziziphus mauritiana* Lam. (BWS-108)	Ber, beri (بیر ،بیری)	Wood, fruit	Digestive disorders, hepatic issues	Edible fruit; laxative (10), increase bile production (6)	Oral	TR	Common	*∗*
*Ziziphus nummularia* (burm. F.) wight and Arn (BWS-109)	Jangli ber (جنگلی بیر)	Fruit, shoots	Nourishment	Edible fruit help in malnutrition (11)	Other	SB	Common	*∗*
Rosaceae/*Rosa alba* L. (BWS-106)	Chitta gulab (چٹہ گلاب)	Flower petals, juice, oil	Antimicrobial, digestive disorders, ornamental, perfumes, food	Rosewater is of medicinal value. It is skin tonic (10), antimicrobial (10) and laxative (10).	Oral	SB	Common	*∗*
*Prunus persica* (BWS-110)	Aru (آڑو)	Leaves, fruit, seeds	Digestive disorders, skin disorders, animals' treatment	Leaves of this plant kill worms (10). Extract of leaves is used to kill worms found in wounds of cattle (11). The ripened fruit is good for the proper functioning of the digestive system (11).	Oral, topical	TR	Common	*∗*
*Rosa indica* L. (BWS-111)	Desi gulab (دیسی گلاب)	Flower, oil	Skin disorders	The paste is used to enhance the skin glow (20)	Oral, topical	SB	Common	[17]*∗*
*Rosa damascena* Mill. (BWS-038)	Gulab (گلاب)	Flower petals, oil	Skin disorders	Petals are used to treat skin disorders (5)	Tropical	SB	Rare	*∗*
*Eriobotrya japonica* (thumb.) Lindl. (BWS-049)	Lokaat (لوکھاٹ)	Fruit	Diabetes	The ripened fruit is edible and the extract is used to treat diabetes (16)	Oral	TR	Common	*∗*
Rutaceae/*Citrus aurantifolia* (christm.) Swingle. (BWS-039)	Nimboo (نمبو)	Fruit	Infections, malaria, fever, cough, skin disorders	Juice of fruit is used in the treatment of fever and malaria (12). Fruit juice and the extract from fruit peel are used to cure acne and black marks on the skin (20). The fruit is used in cosmetics.	Oral, topical	SB	Common	*∗*
*Citrus maxima* (burf.) Merr. (BWS-036)	Chakotra (چکوترا)	Leaves, fruit	Diabetes	Fruit juice is useful for diabetic patients (14)	Oral	SB	Common	*∗*
Scrophulariaceae/*Verbasum thapsus* L. (BWS-037)	Gitthar tambako (گتھر تمباکو)	Leaves	Narcotic, respiratory disorders	The plant is narcotic (4). The smoke of dried leaves is inhaled in bronchitis (3)	Inhaled	SB	Common	
Solanaceae/*Capsicum annuum* L. (BWS-048)	Surkh mirch (سرخ مرچ)	Fruit	Snake bites	Fruit paste is used against bites of insects (8)	Oral, cataplasm	SB	Fruit	*∗*
**† ** *Datura innoxia* Mill. (BWS-042)	Aam dhadura (عام دھاتورا)	Root, stem, leaves, fruit, seeds	Skin disorders	Flower extract is used for the treatment of skin disorders such as itching, scabies, ulcer, leprosy dandruff (4). The plant is poisonous.	Oral	SB	Rare	*∗*
**† ** *Datura metel* L. (BWS-040)	Kala datura (کالا داتورا)	Root, stem, leaves, fruit, seeds	Skin disorders, treatment of rabid dog-bites	Extracts are used for skin treatments such as itching, scabies, ulcer, leprosy dandruff (3). The plant is poisonous. Leave extract is applied on rabid dog-bites (2).	Cataplasm	SB	Common	
*Nicotiana tabacum L*. (BWS-041)	Tambaco (تمباکو)	Leaves	Digestive disorders, narcotic, neural issues, respiratory treatment	Aqueous extracts and tinctures are laxative (8), tonic, emetic (2), narcotic (10), carminative (1), antiseptic (6), sedative (10), and useful in bronchitis and asthma (12). Dried leaves are smoked as narcotics.	Oral, inhaled	SB	Common	*∗*
*Solanum indicum* L. (BWS-043)	Bari kandiari (باری کنڈیاری)	Fruits, seed	Respiratory disorders	Extracts are used for the treatment of catarrhal infections (2). Fruit tea is prepared to cure asthma and cough (8).	Oral	PS	Common	*∗*
*Solanum nigrum* L. (BWS-047)	Makoo, pilk (مکو ،پلک)	Leaves, fruit, seeds	ENT issues, digestive disorders, skin disorders and infections treatment	Root bark extract is a laxative (6), useful in diseases of ears, eyes and nose (2). It is good for ulcers on the neck (2), burning of throats and chronic fever (2).	Oral, topical	HB	Common	[17]*∗*
*Solanum surattense* burm. f. (BWS-046)	Chhoti kandiari (چھوٹی کنڈیاری)	Leaves, fruit, seeds	Influenza, fever, difficult urination, bladder stone, sore throat, cardiac diseases and promote fertility in women.	Plant aqueous extracts are used for the treatment of bladder stones and painful urination (7). Tinctures are prepared to treat influenza, cough (7) and sore throat (9). The fruit extract is considered useful to promote fertility in women (4). The seed extract is used to treat cardiac ailments (2).	Oral	HB	Rare	
*Withania somnifera* (L.) Dunal (BWS-112)	Asgand (اصغند)	Roots, fruit, seeds	Diabetes, insomnia treatment	Leaves and roots are used for restful sleep. The extract is prepared from leaves and roots to treat diabetes (6).	Oral	HB	Common	[17]*∗*
Tamaricaceae/*Tamarix aphylla* (L.) Karst. (BWS-113)	Pilshi (پلشی)	Shoots, wood	Anti-infectious	The smoke of the shoot is antimicrobial (5)	Inhaled	MT	Rare	[17]
Verbenaceae/*∗Vitex negundo* L. (BWS-114)	Bannaa (بانا)	Leaves, young twigs	Respiratory disorders, nervous disorders	Leaves are heated with mustards oil and applied to the chest in case of bronchitis (8). Young twigs are eaten to cure cough (8), asthma (8), fever (4), eye diseases (6), inflammatory (2), intestinal worms (3), ulcers (3), nervous disorders (3) and leprosy (3).	Oral, topical, cataplasm	MT	Common	
*Lantana camara* L. (BWS-045)	Punj phuli (پنج پھولی)	Whole plant	Hepatoprotective	Extracts are used for the treatment of jaundice (3)	Oral	SB	Common	*∗*
Vitaceae/*∗Vitis vinifera* L. (BWS-044)	Angoor (انگور)	Fruit	Cough, digestive disorders	The fruit is nutritive, tonic and medicinal (2)	Oral	LC	Rare	*∗*

Occur, occurrence; Adm, administration; URs, use report; Rpt; reported, HB, herb; SB, shrub; TR, tree; PE, parasitic epiphyte; BT, bushy tree; TT, tall tree; BSH, bushy shrub; MP, medium palm; GH, glabrous herb; HWB, herb woody base; CP, creeping herb; RH, rhizobious herb; MT, medium tree; SH, small herb; SHS, shrub with hallow stem; CLH, cultivated herb; PS, prickly shrub; LC, large climber; CRH, climbing herb; *∗* indicates species enlisted in the IUCN Red List of Threatened Species; † represents poisonous plants, *∗* indicates plants enlisted in Pakistan Herbal Pharmacopoeia. References from previous ethnomedicinal studies from district Sialkot and comparison with Pakistan Herbal Pharmacopeia that reported similar formulations to treat similar ailments are decorated as well.

**Table 3:** Diseases, use report and number of species.

ICPC-2	Disease/action	Use reports	No. Of species
W83	Abortion induced (abortifacient)	10	3
B82	Anemia	42	4
A26	*Cancer*	3	1
K84	Cardiac disorders	16	3
R09	Catarrhal inflation (sinus infections)	10	1
D12	Constipation	63	9
R05	Cough	115	13
S24	Dandruff	10	2
W99	Delivery issues	16	2
D19, D82	Dental ailments	20	3
T89, T90	Diabetes	70	4
D29	Digestive issues	290	32
D07	Dyspepsia	36	4
F73	Eye infections	15	2
A03	Fever/febrile/cold	102	18
A10	Hemorrhage/wounds/stop bleeding	49	8
K86, K87	Hypertension	40	8
F05	Impaired vision	30	1
A08	Inflammation	17	4
A78	Infections (antimicrobial)	95	11
D13	Jaundice	18	5
U14	Kidney stones	46	8
	Leprosy	19	5
D97	Liver issues	65	9
A73	Malaria/dengue	62	5
T91	Malnutrition	28	3
P85	Mental retardation	3	1
N99	Neurological disorders	50	7
A01	Pain reliever (analgesic)	21	5
	Piles	2	1
W17, W18	Postpartum issues/recovery	5	1
R83	Reproductive disorders	54	6
R96	Respiratory disorders/asthma	27	6
L99	Rheumatism	48	3
Y08	Sexual disorders	10	2
	Septicemia (blood purifier)	83	8
S11, S76	Skin infections/disorders	279	27
A77	Small pox	2	1
S12	Snake bites and other stings	39	4
D87	Stomach pain/issues	77	13
U99	UTIs	40	9
D10	Vomiting	2	1
	**Total**	**2029**	**263**

ICPC-2; International *Classification of Primary Care-2*^*nd*^*Edition*.

## Data Availability

The data used to support the findings of this study are included within the article.
